# Local Media Image Propagation Algorithm and Its Governance in the Age of Artificial Intelligence

This article has been retracted.

**DOI:** 10.1155/2022/7723634

**Published:** 2022-02-23

**Authors:** Ming Guo, Weichen Jia

**Affiliations:** ^1^School of Culture and Communication, Guangdong Polytechnic of Science and Technology, Zhuhai 519090, China; ^2^School of Media and Law, Ningbo Tech University, Ningbo, 315000, China

## Abstract

With a large number of images provided by TV and other media flowing into the Internet and the reduction of technical barriers, images have not only become a daily practice for people to record their lives and communicate their behaviors but also become an important means for the public to express their discourse in the cyberspace. Therefore, it is of great significance to analyze the image propagation algorithm using artificial intelligence. This paper mainly studies the algorithm analysis and governance of local media image propagation in the era of artificial intelligence. In this paper, the media is the research object, with its daily dissemination of video works as the research text, in order to discover the ethical problems in its dissemination activities as the purpose, integrating disciplinary knowledge to analyze the ethical problems in this art form, and trying to find out the fundamental measures to solve the problem. The advantages and disadvantages of the video recommendation intelligent algorithm based on the BP neural network are analyzed. By comparing different algorithms, it can be seen that the video recommendation accuracy of the BP neural network algorithm based on swarm optimization (FEBP) is 15.8% higher than that of the traditional BP neural network algorithm. These intelligent algorithms are added into the image transmission system, in order to achieve the goal of improving the image transmission and recommendation effect.

## 1. Introduction

From the perspective of image function, the close relationship between people and image is unparalleled in any period before. While experiencing the charm of digital images through vision and hearing, people's daily life has been bound with numerous digital images, which cannot be easily separated. We cannot imagine how people can survive in today's society without video communication. In today's society, video communication satisfies users' diverse needs of information acquisition, visual enjoyment and entertainment, self-recording and expression, and video art creation. In new media events, the phenomenon of netizens expressing antagonistic words through video transmission is becoming more and more intense. While China is actively building a harmonious society, it is particularly important to guide netizens to the correct expression mechanism of video text in new media events, which is the research background and origin of this paper.

Foreign research on image communication mainly focuses on three aspects: First, it discusses the changes of media events. Secondly, some researchers are committed to emphasizing the role of new media technology in promoting media events. Thirdly, some researchers have explored the relationship between new media and media events in China [1]. The emergence of image production and communication technology makes image-based TV media enter people's daily life, and paper media dominated by text and printing technology has been strongly impacted [2]. Some scholars have creatively established the research theme of iconology in terms of ideology [3]. However, at present, there are few researches on image propagation using artificial intelligence and computer technology. This paper analyzes the image propagation of local media by using BP neural network improvements based on the bee colony algorithm.

This paper studies new media events from the field of visual culture and image communication, studies new media events from different perspectives, and explores the public communication behavior more deeply.

## 2. Image Propagation Algorithm Analysis and Its Governance

### 2.1. Image Propagation Type

At present, microvideo content providers mainly include traditional TV stations, commercial websites, professional film and television production institutions, and citizen creation. Due to the great attention of all parties to social media, they participate in the production of microvideos in different ways.

#### 2.1.1. Traditional Media

Traditional media have the natural conditions to create microvideos, because they have the unique right to interview and broadcast and also have the professional foundation of film and television creation. Variety shows, news videos, sports broadcasts, and entertainment programs produced by traditional media also provide material reserves for microvideos and become important content sources for social media to provide on-demand services [4]. With the spread of Internet technology, traditional media have tried the waters with microvideos. For example, the Beijing News' “Moving News” videos, each of which is only three minutes long, were created with the integration of modern video technology, reducing the ethical and technical problems posed by traditional videos. However, the insensitivity of the communication mechanism is also a shortcoming of traditional media in the march of microvideo communication.

#### 2.1.2. Network Media

In the Internet era, all kinds of commercial portal websites have won a large number of traffic and users based on the transmission of images. At present, they are also actively turning to the microend. Video websites of various types also play an important role in microvideos on mobile Internet, relying on their experience, user stickability, and reputation in operating video content accumulated in fixed network and PC terminals. They mainly cooperate with CP of communication operators to expand the spread of website content in social media [5]. News and information, entertainment and variety shows, and animation and games produced by video websites are also important content sources. And it will be shared on social media in time to further expand the influence of the program.

#### 2.1.3. Professional Film and Television Production Organizations

With the increase of China's economic openness and the further development of the diversification of market subjects, a large amount of private capital began to inject into the cultural media industry. Compared with traditional media, it has an independent legal personality. Different from commercial websites, these professional cultural media companies generally do precise and niche content marketing. They are the main producers of TV series, films, column short films, movie trailers, movie tidbits, and TV drama trailers, etc. Now, most of them are private enterprises [6]. There are organizations that specialize in video production for social media, and they produce short videos with some sort of continuity or reintegration of microvideo content that will be better suited to social media platforms.

#### 2.1.4. Netizen Uploading

Users include individual uploads by netizens, who refer to individual uploads by network users or social media users. That is to say, as long as they have the equipment, people may become the providers of works. Netizens have so many sources of information that they can take photos of news events anytime and anywhere and upload them online without screening them. At present, videos shot by netizens themselves have become the mainstream of microvideos on social media. The video works forwarded by netizens have become the main source of social media video transmission. The cultural media team produces different works, and most of the videos made by netizens are spontaneous, original, and time-sensitive.

### 2.2. Governance Strategies for Image Communication Issues

The social regulation means of mass media include the public power in mass media activities, mass media literacy education and media content classification systems, and other related contents. The image communication of social media is a part of mass media. How to solve the problems arising from social media should not only rely on the guidance and constraints of the state. Self-discipline and regulation of the industry need greater participation and consciousness of the whole people.

#### 2.2.1. Improve Relevant Laws and Regulations

As for the problem of infringement in the transmission of social media images, we have not formed special laws and regulations to govern. Take the United States as an example; the government of the United States promulgated the Privacy Law as early as the 1970s, which can be regarded as the basic law of privacy protection. In contrast, there is no independent privacy protection law in China. The United States protects the privacy of its citizens quite well, and even though social media is developing rapidly, it still needs to be guided by the law. On social media, privacy can easily be exposed and even litigated. The experience of foreign countries should be used for reference, and the privacy of citizens should be strictly protected. There will always be problems in the dissemination of images on social media. If we follow the steps to deal with these problems, they cannot be fundamentally solved. Therefore, the formulation of national laws and regulations needs to be forward-looking and flexible.

#### 2.2.2. Improve Industry Supervision Technology

Technology update lacks effective supervision over media communication content. Despite media violence or bad media information, currently, Chinese laws have no clear definition and description of vulgar information. Although people hope to strengthen active supervision, long-term supervision has not been implemented. First, because of the concealment of information, the spread of a wide range of regulatory technology may not be able to keep up, and vulgarity is a concept of no legal significance, only from the moral explanation. There are certain regional and temporal differences. The rectification of media vulgarity encountered a bottleneck; the regulatory departments brought difficulties and obstacles but also made bad media opportunities. On the one hand, the updating technology should grasp the development trend and direction of self-regulation technology, such as filtering software should be developed toward intelligent filtering and deep filtering, hierarchical filtering technology should give end users maximum autonomy, and hierarchical filtering systems should realize interoperability and compatibility among other functions.

#### 2.2.3. Improve the Ways of Image Communication Literacy

It is of great significance to study and grasp the aesthetic value of microvideos. It is conducive to enhancing people's understanding of the aesthetics of microvideos, guiding and promoting the recording subject and receiving assistant's pursuit of the aestheticization of microvideo works and conducive to the degree of grasp and showing new degrees. Excellent micro video works should be the product of seeking new things. Record and report new things, new themes, new understanding, the pursuit of new angles, new forms, and new skills. It is necessary to improve the ability of media cognition, criticism, and utilization. In the discussion of the technology gap, it has been shown that Internet technology will widen the knowledge gap, making the rich richer and the poor poorer. In a sense, we must improve the media literacy of users so that they can distinguish the right and good things and discard the wrong and bad things.

### 2.3. Image Propagation Algorithm

#### 2.3.1. BP Neural Algorithm

The BP neural network is mainly composed of three layers, the input layer (S), the hidden layer (a), and the output layer (R), in which the input layer, hidden layer, and output layer are composed of several similar neurons, each layer of BP neural network is linked by neurons. The images for this article are drawn by Visio. The input layer is used for the input of the feature vector, the hidden layer is used for the hidden neural layer in the network, and the output layer is used for the output of the network algorithm [7, 8].

The flow chart of the BP neural network algorithm is shown in Figure 1.

If there are *N* training samples, for each neuron, the training error of each training sample in this neuron can be expressed as

(1) $$\begin{array}{c} \text{Er}=\frac{1}{2}\overset{L}{\underset{c=1}{\sum }}\overset{n_{c}}{\underset{j=1}{\sum }}{\left(y_{cj}-\bar{y_{cj}}\right)}^{2}, \end{array}$$

where *n*_*c*_ represents the number of neurons at each layer in the neural network (NeNt), *L* represents the number of corresponding layers, and *y*_*cj*_ represents the actual output value. Therefore, for all training samples, the total error of the NeNt algorithm can be expressed as

(2) $$\begin{array}{c} E=\frac{1}{2}\overset{N}{\underset{r=1}{\sum }}\text{E}\text{r}. \end{array}$$

Through this training error, BPNN continuously adjusts and corrects the connection weights between each layer of neurons in the NeNt algorithm until the total error of the algorithm is reduced to an acceptable level. The formula for correcting the connection weights is as follows:

(3) $$\begin{array}{c} w_{ij}=w_{ij}-\mu \frac{\partial E_{r}}{\partial w_{ij}}, \end{array}$$

where *μ* is the learning rate and *w*_*ij*_ is the connection weight between neuron *i* and neuron *j*.

The main steps of using the NeNt algorithm for classification are as follows: data normalization, creation of NeNt, training of NeNt, and classification of NeNt. The NeNt algorithm can effectively solve the nonlinear and variable sample classification problem [9, 10].

#### 2.3.2. BPNN Algorithm Based on Bee Colony Optimization

The BPNN algorithm based on colony optimization (FEBP algorithm) adopts the idea of the swarm intelligence algorithm. Through the principle of hiring bees, observing bees, and reconnaissance bees to search for the nectar source, in-depth research is carried out, and the idea of searching for the nectar source by bees is integrated into the BPNN.

The iterative idea of the bee colony intelligent algorithm is used to initialize the optimal weights and thresholds of the nodes of each layer of the BPNN, which reduces the iterative optimization time of the BPNN and reduces the risk of the BPNN falling into the local optimum. The weights and thresholds of the BPNN will be continuously updated, so that the error of the BPNN reaches the set threshold, thereby terminating the algorithm.

The BPNN based on bee colony optimization has the advantages of high precision, small error, and fast convergence, which can effectively solve the historical problem of BPNN being trapped in a local optimal solution. By applying the BPNN algorithm based on bee colony optimization in the video recommendation system, it can have a better video recommendation effect and improve user perception.

The BPNN algorithm based on bee colony optimization mainly includes two processes: the principal component analysis (PCA) reduces the dimensionality of sample collection, and the main components are used to replace the original data set; secondly, the swarm intelligence algorithm is used to optimize the weights and thresholds to obtain the optimal weights and thresholds, so as to prevent the problems caused by the random option values and thresholds of BPNN.

Common BPNN optimization algorithms include genetic algorithm and particle swarm optimization algorithm. The genetic algorithm is suitable for solving discrete problems, but there is the Hamming cliff problem; particle swarm optimization (PSO) is suitable for solving real number problems. The algorithm is simple, but there are local optimal problems. However, using the bee colony algorithm to optimize BPNN and find the optimal network weights and thresholds can have both the generalization mapping ability of NeNt and the characteristics of global iteration and local search of bee colony algorithm, so it has better optimization effect compared with other algorithms [11].

## 3. Algorithm Simulation Experiment

### 3.1. Experimental Process

This paper mainly uses the Python tool language for raw data processing, algorithm implementation, and experiments and uses MATLAB tools to compare and analyze the experimental results. The Python language is an object-oriented interpretive computer language, with powerful libraries, such as machine learning library skearn-learn and convenient developers to complete all kinds of programs; it has powerful visualization function and is suitable for the comparative analysis of the experimental results.  Table 1 shows the computer experiment environment of this paper.

### 3.2. Experimental Data

This section mainly introduces the BPNN video recommendation algorithm based on bee colony optimization. The MovieLens 1M data set is adopted in the experiment, which includes the user data set, video data set, and user's video rating data set; these three data sets were combined using Python tools to obtain a data set containing user ID, video ID, user age, user gender, video type, and user rating of the video. Then, feature extraction is carried out on this data set, and the principal component feature set of the user's video rating is finally obtained through calculation, as shown in Table 2.

### 3.3. Evaluation Index of Algorithm Experiment

In order to effectively verify the effectiveness of the experimental results of the BPNN video recommendation algorithm based on bee colony optimization and compare the recommendation performance of different algorithms, it is necessary to evaluate the recommended output value and the true value of the algorithm. Commonly used methods to evaluate the classification performance of algorithms are accuracy, mean square error (MSE), confusion matrix, cross-entropy loss function, accuracy, recall, etc. This paper uses precision, mean square error, cross-entropy loss function, correct rate, recall rate, and F1_score to evaluate each algorithm.

## 4. Comparison and Analysis of Experimental Results

### 4.1. Algorithm Accuracy Comparison

Accuracy mainly reflects the accuracy of the algorithm in sample classification. The closer the classification result is to the real result, the greater the value of the accuracy will be, and the better the accuracy of the algorithm will be. As shown in Table 2 and Figure 2, the accuracy of the FEBP algorithm in the classification of user ratings is higher than that of the traditional BP algorithm and GA-BP algorithm. The video recommendation accuracy of the BPNN algorithm based on the bee colony optimization (FEBP) is 15.8% higher than that of the traditional BPNN algorithm. In the case of a relatively small test sample set, the BPNN algorithm based on colony optimization has a lower accuracy than GA-BP algorithm. However, with the continuous increase of sample tests, the classification accuracy of the BPNN algorithm based on colony optimization for the video score is continuously improved compared with the BP and GA-BP algorithms.

### 4.2. Algorithm Mean Square Error Comparison

The mean square error can qualitatively judge the mean error of the algorithm in the classification of the sample set. The smaller the mean square error is, the lower the sample classification error is. As shown in Table 3 and Figure 3, compared with the traditional BPNN algorithm and the GA-BP algorithm, the equipartition error is reduced to different degrees. After that, based on swarm optimization of BPNN to classification video score has lower average error than other algorithm. But just judging from the accuracy rate and mean square error (mse), FEBP algorithm for video rating classification is persuasive enough; better accuracy and mean square error (mse) algorithmn can explain the overall classification precision high; in the real network, the user's rating of videos is a subjective and personalized event, so more refined indicators are needed to test the user rating classification algorithm.

### 4.3. Comparison of FER Values of the Algorithm

Based on the knowledge of the neural network algorithm, the cross-entropy loss function is used to measure the robustness of the algorithm. The experimental results of the cross-entropy loss function of each algorithm in the recommendation system based on user ratings and video types are shown in Table 3.

In this paper, the F1_score, precision, and recall are used to evaluate the recommendation effect of the recommendation system. As shown in Figure 4, the BPNN algorithm based on bee colony optimization has better accuracy, recall rate, and F1_score than the traditional BPNN and GA-BP algorithms for the videos that users are interested in (the videos with scores ≥ 4 are the videos that users are interested in).

## 5. Conclusions

This is a new era of video communication; we need to face up to the ethical anomie problem of video communication and explore the way to correct the deviation from the existing ethical thoughts. Deontological thinking urges us to self-examine and strengthen self-discipline from our own perspective. Utilitarianism, on the other hand, reminds us to start from the maximal happiness of the greatest number of people and strengthen the “double insurance” of heteronomy. Good image communication environment and network ecology are related to a country's economic, political, cultural, and other aspects of development but are also related to the future of a nation, which require the joint efforts of the government, platform, and many users. There is still a long way to go to solve the problem of anomie in video communication ethics. Therefore, this paper puts forward suggestions from the government, mainstream media, and the public to promote rational discourse expression of image communication in new media events. First of all, the government should make information transparent, win the trust of the public, eliminate the misunderstanding between the government and the people through dialogue and communication, rebuild the social trust mechanism, and promote the resolution of the discourse conflict between the government and the people. Secondly, when reporting new media events, mainstream media should provide comprehensive and objective information, weaken visual conflicts, objectively report facts, safeguard the interests of the public, and strengthen the guidance of mainstream values. Finally, the public should start from their own, enhancing social responsibility, improving visual recognition ability, and promoting rational discourse expression.

## Figures and Tables

**Figure 1:** Flow chart of BP neural network algorithm.

**Figure 2:** Comparison of accuracy of different algorithms.

**Figure 3:** Algorithm mean square error comparison.

**Figure 4:** Algorithm FPR value comparison.

**Table 1:** System development environment.

CPU	Intel Core i510400
Memory	16 GB
Graphics card	NVIDIA RTX2060
Operating system	Windows 10

**Table 2:** Each principal component of the characteristic data set.

Principal components	Contribution	Cumulative contribution rate
Video ID	14.9%	14.9%
Main type of video	19.4%	34.3%
Video subtype	16.7%	51.0%
User age	23.1%	74.1%
Number of male users	7.3%	81.4%
Number of female users	8.7%	90.1%

**Table 3:** Algorithm cross-entropy loss function.

Algorithm	BP algorithm	GA-BP	FEBP
Cross-entropy	0.2753	0.2682	0.2417

## Data Availability

The data underlying the results presented in the study are available within the manuscript.
